The article "IAA8 Involved in Lateral Root Formation Interacts with the TIR1 Auxin Receptor and ARF Transcription Factors in Arabidopsis" was published in 2012. Journal: PLoS One.

# IAA8 Involved in Lateral Root Formation Interacts with the TIR1 Auxin Receptor and ARF Transcription Factors in *Arabidopsis*

**DOI:** 10.1371/journal.pone.0043414

**Published:** 2012-08-17

**Authors:** Fumi Arase, Hiroko Nishitani, Mayumi Egusa, Nami Nishimoto, Sumiko Sakurai, Naho Sakamoto, Hironori Kaminaka

**Affiliations:** Laboratory of Plant Molecular Biology, Faculty of Agriculture, Tottori University, Tottori, Japan; Instituto de Biología Molecular y Celular de Plantas, Spain

## Abstract

The expression of auxin-responsive genes is regulated by the TIR1/AFB auxin receptor-dependent degradation of Aux/IAA transcriptional repressors, which interact with auxin-responsive factors (ARFs). Most of the 29 *Aux/IAA* genes present in *Arabidopsis* have not been functionally characterized to date. *IAA8* appears to have a distinct function from the other *Aux/IAA* genes, due to its unique transcriptional response to auxin and the stability of its encoded protein. In this study, we characterized the function of *Arabidopsis IAA8* in various developmental processes governed by auxin and in the transcriptional regulation of the auxin response. Transgenic plants expressing estrogen-inducible *IAA8* (*XVE::IAA8*) exhibited significantly fewer lateral roots than the wild type, and an *IAA8* loss-of-function mutant exhibited significantly more. Ectopic overexpression of *IAA8* resulted in abnormal gravitropism. The strong induction of early auxin-responsive marker genes by auxin treatment was delayed by *IAA8* overexpression. GFP-fusion analysis revealed that IAA8 localized not only to the nucleus, but, in contrast to other Aux/IAAs, also to the cytosol. Furthermore, we demonstrated that IAA8 interacts with TIR1, in an auxin-dependent fashion, and with ARF proteins, both in yeast and *in planta.* Taken together, our results show that IAA8 is involved in lateral root formation, and that this process is regulated through the interaction with the TIR1 auxin receptor and ARF transcription factors in the nucleus.

## Introduction

Auxin was the first phytohormone to be discovered and is well-known for its regulatory role in various developmental processes, such as growth and differentiation, and in the cellular responses to light, phosphate starvation, and pathogens [1], [2]. The versatile nature of auxin molecules seems to stem from the complex regulation of auxin metabolism, transport, signaling, and response. The binding of an auxin molecule to TIR1 (TRANSPORT INHIBITOR RESPONSE 1) and AFB (AUXIN F-BOX PROTEIN) receptor proteins is the cue for the transcription machinery to induce auxin-responsive genes [3]–[5]. TIR1/AFB proteins, F-box proteins that form part of the SCF ubiquitin-ligase complex (SCF^TIR1/AFB^) [6]–[8], target Aux/IAA (AUXIN/INDOLE-ACETIC ACID) transcriptional repressors for ubiquitin-mediated degradation [8]–[11]. Aux/IAA proteins block the activity of ARF (AUXIN RESPONSE FACTOR) transcription factors by forming a heterodimer with this molecule when the cellular level of auxin is low [5]. The degradation of Aux/IAA proteins by SCF^TIR1/AFB^-mediated ubiquitination following the perception of auxin molecules promotes ARF-mediated transcription. Therefore, the dynamic changes in Aux/IAA abundance, which are controlled by cellular auxin levels, determine the expression levels of auxin-responsive genes.

*Aux/IAA* genes, which were initially identified as a large family of early auxin-response genes [12], are unique to plants and encode unstable nuclear proteins with four conserved domains [13]. Domain I contains an ERF-associated amphiphilic repression (EAR)-motif, which allows the Aux/IAA protein to interact with the co-repressor protein TOPLESS (TPL) and TPL-related (TPR) proteins [14]. Domain II is recognized by the SCF^TIR1^ complex and is involved in the instability of Aux/IAA proteins [15], [16]. Domains III and IV mediate both the homodimerization of Aux/IAA proteins and their heterodimerization with ARF proteins [13], [17], [18]. The *Arabidopsis* genome encodes 29 Aux/IAA proteins [19]. Numerous functional analyses of *Aux/IAA* genes have been conducted by molecular and biochemical methods and by characterization of mainly gain-of-function mutants. Analysis of proteolytic degradation using transiently expressed Aux/IAA-luciferase fusions suggested that significant primary sequence and structural variations in the receptor recognition motif within domain II affect the stability and longevity of Aux/IAA proteins treated with auxin [20]. Gain-of-function mutations within domain II, which stabilize Aux/IAA proteins, have been found in independent mutant screenings based on altered auxin response or morphology [13], whereas loss-of-function mutations in *Aux/IAA* genes have little effect on the phenotype [19]. The functional analysis of plants with these gain-of-function mutations has demonstrated that *Arabidopsis* Aux/IAAs regulate various developmental processes that are governed by auxin molecules, including gravitropism, lateral root formation, and root and stem elongation [21]–[27]. Although the functions of some of the *Arabidopsis Aux/IAA* genes have been clarified, most of the 29 *Aux/IAA* genes have not been functionally characterized to date.

*IAA8* appears to have a distinct function from other *Aux/IAA* genes; unlike other *Aux/IAA* genes, the expression of *IAA8* is not altered by auxin treatment in various tissues, and IAA8 is more stable than the well-characterized Aux/IAA proteins, IAA1 and IAA17 [12], [20], [28]. Using promoter-GUS transgenic plants, it has been reported that *IAA8* is expressed in the developmental vasculature of the shoot apex, hypocotyl, and root tip, and is developmentally regulated [29]. In this study, we focus on the role of *Arabidopsis* IAA8 in the transcriptional regulation of the auxin response as well as on the control of root development. We have also analyzed the subcellular localization of IAA8 and carried out a comprehensive interaction analysis of IAA8 with its functional partners, the TIR1 auxin receptor and ARF transcription factors. We found that IAA8 regulates lateral root formation and operates as a transcriptional repressor of the auxin response. Interestingly, although IAA8 physically interacts with both TIR1, via an auxin molecule, and ARF proteins, as do other Aux/IAA proteins, its subcellular distribution is distinct.

## Results

### *IAA8* is involved in root development

To characterize the function of *IAA8* in *Arabidopsis*, we generated transgenic plants that overexpress *IAA8*. Initially, we used the Cauliflower Mosaic Virus (CaMV) 35S promoter for the overexpression; however, strong overexpression of *IAA8* in any transgenic plants could not be confirmed (data not shown). Therefore, the estradiol-inducible promoter XVE in the pER8 vector [30] was used to create transgenic plants that conditionally and strongly express *IAA8* (*XVE::IAA8*). The expression of *XVE::IAA8* transgenes upon induction with estradiol was examined in over 20 transgenic lines by semi-quantitative reverse transcriptase-PCR (RT-PCR) analysis. Of *XVE::IAA8* plants examined, *IAA8* expression was induced above endogenous levels only in lines #8 and #11 following estradiol treatment (Figure 1, data not shown).

**Figure 1:** *IAA8* overexpression suppresses the auxin-inducible expression of early auxin-responsive genes in roots. Wild-type (Col-0) and XVE::IAA8 (line #8, #11) roots treated first with 10 μM β-estradiol for 24 h and then with 1 μM IAA for 0 to 60 min were subjected to semi-quantitative RT-PCR analysis of the auxin marker genes, *IAA1*, *IAA19* and *GH3.3* together with endogenous *IAA8* gene expression (end) and of both endogenous and exogenous (end + exo) *IAA8* gene expression. EF1α was used as an internal control. All semi-quantitative RT-PCR figures are representative of three biological replicates.

These *XVE::IAA8* plants were used for further experiments together with a loss-of-function T-DNA insertion mutant of *IAA8*, *iaa8-1* [19]. The aerial parts of *iaa8-1* and *XVE::IAA8* plants did not show any obvious phenotypic change compared with those of wild-type Col-0 plants (data not shown). The absence of visible developmental defects in a loss-of-function mutant of *IAA8* is consistent with findings of a previous report [19].

Since several *Aux/IAA* genes are involved in auxin-related root development, such as primary root elongation, lateral root formation, and grapitropism [21], [22], [24]–[27], [31], we decided to examine these auxin-related root phenotypes in *iaa8-1* and *XVE::IAA8* plants. On normal MS medium, the phenotype of all of the genotypes examined was unaffected (Figure 2A, left; data not shown). Following estradiol treatment, the roots exhibited growth defects, even in Col-0 seedlings (Figure 2A, right). The seedlings of both *XVE::IAA8* lines treated with estradiol exhibited abnormal gravitropism and had more severe root growth defects than estradiol-treated Col-0 plants (Figure 2A, right). However, there was not a statistically significant difference in primary root growth between Col-0 and any of the genotypes treated with estradiol (Figure S1). In contrast, the number of lateral roots in both *iaa8-1* and one of estradiol-treated *XVE::IAA8* plants (line #11) was altered (Figure 2B). A significant increase in the number of lateral roots was observed in *iaa8-1* as compared with Col-0 (Figure 2B, Figure S2), whereas the number of lateral roots in one of estradiol-treated *XVE::IAA8* plants (line #11), which displayed a strong abnormal root phenotype (Figure 2A, right), was reduced (Figure 2B). In addition, the gravitropic response of estradiol-treated *XVE::IAA8* plants was also diminished, whereas that of *iaa8-1* was unaltered as compared with Col-0 (Figure 2C).

**Figure 2:** Effects of loss-of-function and overexpression of *Arabidopsis IAA8* on root phenotypes in seedlings. (A) Effects of estradiol treatment on the phenotype of wild-type (Col-0) and *XVE::IAA8* (line #8 and #11) seedlings. All seedlings were vertically grown for 14 days on 1/2 MS medium containing 10 μM β-estradiol (+β-estradiol) or 0.1% ethanol (−β-estradiol). Bar  = 1 cm. (B) The number of lateral roots was counted on Col-0, *XVE::IAA8,* and *iaa8-1* seedlings grown for 14 days on 1/2 MS medium containing 10 μM β-estradiol (+β-estradiol) or 0.1% ethanol (−β-estradiol). Averages of at least 20 seedlings ± S.D. are shown. A statistical analysis was performed using Student's *t* test, with significant differences indicated relative to Col-0 (* P<0.05, ** P<0.01). (C) Gravitropic response of Col-0, *XVE::IAA8,* and *iaa8-1* seedling roots. Seedlings were grown vertically for 5 days on 1/2 MS medium containing 10 μM β-estradiol, and then reoriented by 90° and grown for 4 days on the same medium. The deviation from a vertical line observed in the primary root growth was measured and assigned to one of twelve 30° sectors in the circular histograms. The length of each bar represents the percentage of seedlings showing the same direction of root growth. Over 30 seedlings were evaluated for each genotype.

### IAA8 suppresses the early induction of auxin-responsive genes

Aux/IAA proteins possess a potent transcriptional co-repression activity through their domain I, which contains an EAR-motif for interaction with the co-repressor protein TPL [14], [32]. A recent interactome study revealed that *Arabidopsis* IAA8 interacts with TPR2, which is one of five TPL/TPR proteins [33]. To determine whether IAA8 also functions as a co-repressor of transcriptional regulation for the auxin response, as do the other Aux/IAA proteins, we examined the effects of *IAA8* overexpression on the induction of early auxin responsive genes using *XVE::IAA8* plants by semi-quantitative RT-PCR analysis. The early induction of three auxin-responsive marker genes (*IAA1, IAA19* and *GH3.3*) [28] by Indole-3-acetic acid (IAA) treatment in roots was suppressed in estradiol-pretreated *XVE::IAA8* plants, especially in line #11, which show drastic changes in root phenotypes (Figure 2), as compared with the wild type (Figure 1).

### The subcellular localization of IAA8 is distinct from that of other Aux/IAA proteins

Aux/IAA proteins generally possess a nuclear-localization sequence (NLS) and are localized to the nucleus [18], [23], [34]–[37]. We used a polyethylene glycol (PEG)-mediated transient expression system in *Arabidopsis* mesophyll protoplasts to determine the subcellular localization of GFP fusions of IAA8, which functions as a transcriptional repressor (Figure 1), and also of the well-characterized Aux/IAA proteins, *Arabidopsis* IAA7 and IAA17. NLS-tdTomato, a nuclear marker consisting of a fusion of simian virus 40 (SV40) large T antigen NLS [38] and red fluorescent protein tdTomato, was co-expressed with the GFP fusions in protoplasts. IAA7-GFP and IAA17-GFP localized exclusively to the nucleus, as previously reported [18], whereas IAA8-GFP localized to both the nucleus and the cytosol (Figure 3).

**Figure 3:** Subcellular localization of IAA7, IAA8, and IAA17. GFP fusions of IAA7, IAA8, and IAA17 were transiently expressed in *Arabidopsis* mesophyll protoplasts. NLS-tdTomato was co-introduced both as a nuclear marker and as a control for transformation. GFP, NLS, and BF (top) represent GFP and tdTomato fluorescence and bright field images, respectively. n: nucleus, c: cytosol. Bars  = 10 μm.

### IAA8 interacts with auxin receptor TIR1 in an auxin-dependent fashion

A key event in the transcriptional regulation of the auxin response is the degradation of Aux/IAA proteins that have been ubiquitinated by TIR1/AFB auxin receptors activated by direct binding to auxin [4]–[6], [8]–[11]. Recently, the auxin-dependent protein-protein interaction between TIR1/AFB receptors and Aux/IAA proteins has been assayed using a yeast two-hybrid system [39]. Therefore, we next performed a yeast two-hybrid assay to examine the auxin-dependent interaction between TIR1 and IAA8. The well-characterized Aux/IAA proteins, IAA7 and IAA17, were used as positive controls for this experiment. In yeast, IAA8, IAA7, and IAA17 interacted with TIR1 only on medium containing IAA (Figure 4A), as previously described for IAA7 and IAA17 [39]. To examine a possible auxin-dependent interaction between TIR1 and IAA8 *in planta*, we further conducted bimolecular fluorescence complementation (BiFC) assays using a transient expression system in *Arabidopsis* mesophyll protoplasts as described above. The N terminal of IAA8 was fused to the N-terminal half of YFP (nYFP) to yield nYFP-IAA8, and the N terminal of TIR1 was fused to the C-terminal half of YFP (cYFP) to yield cYFP-TIR1. The nYFP-IAA7 and nYFP-IAA17 fusions were used as positive controls and nYFP-GUS was used as a negative control. In the negative control experiment using nYFP-GUS and cYFP-TIR1, no YFP fluorescence was observed. Similarly, protoplasts expressing both nYFP-IAAs and cYFP-TIR1 did not show any fluorescent signal in the absence of IAA (Figure 4B, left). In contrast, auxin treatment resulted in strong YFP fluorescence in protoplasts expressing all of the nYFP-Aux/IAA fusions and cYFP-TIR1. This finding corroborated the auxin-dependent interaction between TIR1 and IAA8 as well as IAA7 and IAA17 *in planta* (Figure 4B, right). The YFP fluorescence resulting from the interaction between TIR1 and Aux/IAA proteins in BiFC assays was present only in the nucleus.

**Figure 4:** Auxin-dependent interaction of IAA8 with the TIR1 auxin receptor. (A) Yeast (EGY48::pJK103) cells were co-transformed with bait plasmid, which contained a LexA DNA-binding domain (BD)-TIR1 fusion (BD-TIR1) in pEG202, and prey plasmid, which contained activation domain (AD)-Aux/IAA fusions (AD-Aux/IAA) in pJG4-5. Auxin-dependent interactions in each transformant were assayed by plating on SD(Gal)/-Ura/-His/-Trp/-Leu medium with 100 μM IAA (+IAA). Auxin-independent interactions were examined using the same medium without IAA (−IAA). (B) The BiFC assay was used to detect protein-protein interactions between Aux/IAA repressors and TIR1. *nYFP-Aux/IAA* fusions or *nYFP-GUS* and *cYFP-TIR1* were transiently co-expressed in *Arabidopsis* mesophyll protoplasts with a nucleus marker plasmid, NLS-tdTomato. To monitor the auxin-dependent interaction, 10 μM IAA was added before microscopic observation (+IAA). BiFC, NLS and BF (top) represent YFP, tdTomato fluorescence, and bright field images, respectively. n: nucleus. Bars  = 10 μm.

### IAA8 interacts with ARF transcription factors

The expression of auxin-responsive genes is directly controlled by the transcriptional activity of ARF transcription factors [5]. Five of the 23 ARF proteins present in *Arabidopsis* function as transcriptional activators, whereas the remaining eighteen act as repressors [32]. At low auxin levels, ARF transcriptional activity is blocked by direct interaction with Aux/IAA proteins. Increased cellular levels of auxin result in the degradation of Aux/IAA proteins that have been ubiquitinated via their interaction with TIR1/AFB receptors and thereby promote ARF transcriptional activity [5]. The heterodimerization of Aux/IAA and ARF proteins occurs via an interaction between the conserved domains III and IV on both proteins [18], [25], [27], [40]. To clarify whether IAA8 interacts specifically with ARFs, we carried out another series of yeast two-hybrid and BiFC analyses. The semi-quantitative *lacZ* activity assays used to measure the protein-protein interaction levels in the yeast two-hybrid system showed that IAA8 strongly interacted with the C-terminal domain (CTD), which contains domain III and IV, of the ARF activators, ARF5, ARF7, and ARF19 (Figure 5A). The *lacZ* activity for ARF3, which does not contain domain III and IV, was almost the same as in the negative control experiment (Figure 5A). On the other hand, ARF4, ARF11, and ARF16, which are ARF repressors that contain domain III and IV, directly interacted with IAA8. However, the level of this interaction was much lower than that of the ARF activators (Figure 5A). Western blot analysis of AD-ARFCTD proteins using anti-HA antibody reveals that the expression level of each ARF protein in yeast does not affect the intensity of interaction with IAA8 (Figure S3).

**Figure 5:** Detection of the interaction between IAA8 and ARFs by yeast two-hybrid and BiFC assays. (A) Yeast (EGY48::pJK103) cells were co-transformed with BD-IAA8 bait plasmid and AD-ARFCTD prey plasmid as in Figure 4. The strength of each interaction was evaluated by measuring β-gal activity using the o-nitrophenyl β-D-galactopyranoside (ONPG) method. Vector indicates empty vector (negative control experiment). (B) A BiFC assay was carried out to monitor the protein-protein interaction between IAA8 and ARFs. *ARF-nYFP* fusions or *nYFP-GUS* and *IAA8-cYFP* were transiently co-expressed in *Arabidopsis* mesophyll protoplasts with a nuclear marker plasmid, NLS-tdTomato. BiFC, NLS, and BF (top) represent YFP, tdTomato fluorescence, and bright field images, respectively. n: nucleus. Bars  = 10 μm.

To further analyze the *in planta* protein-protein interaction between Aux/IAA proteins and ARFs, we performed a BiFC analysis by transiently expressing ARF-nYFP fusions, the C-terminal fusion of ARF with nYFP, and IAA8-cYFP, the C-terminal fusion of IAA8 with cYFP, in *Arabidopsis* mesophyll protoplasts. The negative control experiment using nYFP-GUS and IAA8-cYFP did not result in any YFP fluorescence (Figure 5B). As expected, protoplasts expressing both ARF3-nYFP and IAA8-cYFP also lacked YFP fluorescence, because ARF3 lacks domain III and IV [19]. Using all other ARF-nYFP/IAA8-cYFP combinations, strong YFP fluorescence derived from specific physical protein-protein interactions was observed only in the nucleus (Figure 5B).

## Discussion

### *IAA8* is involved in lateral root formation

Most of 29 *Aux/IAA* genes present in *Arabidopsis* have not yet been functionally characterized. Of the poorly characterized *Arabidopsis Aux/IAA* genes, *IAA8* was predicted to have a distinct function from the other *Aux/IAA* genes, based on its different transcriptional response to auxin and protein stability [12], [20], [28]. In this study, we first analyzed the phenotypes of transgenic plants that conditionally overexpressed *IAA8*, *XVE::IAA8,* and an *IAA8* loss-of-function mutant, *iaa8-1* [19], to clarify the function of IAA8 in various developmental processes governed by auxin. No developmental defects in aerial parts were observed in any of the *IAA8* plants studied (data not shown). Since gain-of-function mutations in several *Aux/IAA* genes alter auxin-related root development [21], [22], [24]–[27], [31], we examined the root phenotypes of the *IAA8* plants. Although primary root lengths were normal for all of the genotypes examined (Figure S1), there was a significant difference in the number of lateral roots and in the gravitropic response (Figure 2). Abnormal gravitropism was only found in the plants that ectopically overexpressed *IAA8* and not in the loss-of-function mutant. Similar phenotypic changes were also observed in plants that overexpressed the non-canonical *Aux/IAA* genes, *IAA20*, *IAA30,* and *IAA31* [41]. The half-lives of the non-canonical Aux/IAA proteins, which lack or partially lack domain II, are much longer than those of canonical Aux/IAAs, like IAA17 [20]. Considering that the half-life of IAA8 is also longer than that of other well-characterized Aux/IAA proteins [20], the gravitropic response appears to be affected by the ectopic overexpression of *Aux/IAA* genes that encode relatively stable proteins.

In contrast, the number of lateral roots was altered in *XVE::IAA8* and *iaa8-1* plants, being decreased in the former and increased in the latter (Figure 2). Thus, *IAA8* appears to be involved in lateral root formation. However, the phenotypic changes in lateral root formation in *XVE::IAA8* and *iaa8-1* were distinctly weaker than those observed in other *Aux/IAA* gain-of-function mutants (e.g., *shy2/iaa3*, *slr-1/iaa14*, *crane/iaa18,* and *msg2/iaa19*) [22], [25]–[27]. This discrepancy could be due to differences between overexpression and dominant gain-of-function mutations of *Aux/IAA* genes. In dicots, including *Arabidopsis*, lateral root initiation depends on the activation of pericycle cells by auxin [2]. *IAA8* promoter-driven *GUS* expression is found in the vascular tissue of the root tip, which appears to correspond to pericycle cells [29], but *IAA8* is not up-regulated by auxin [12]. In lateral root formation, therefore, IAA8 seems to participate in the transcriptional regulation of the auxin response together with other Aux/IAA proteins involved in lateral root formation; however, its expression and function might be regulated by a signaling pathway not governed by auxin.

### IAA8 is a transcriptional repressor of the auxin response in the nucleus, but is potentially imported into the cytosol

Aux/IAA proteins interact with the co-repressor protein TPL via the EAR-motif in domain I to exert potent transcriptional co-repression [14]. As expected, the strong induction of early auxin responsive marker genes by auxin was delayed by *IAA8* overexpression (Figure 1). A recent report revealed that IAA8 interacts with one of five TPL/TPL-related (TPR) proteins, TPR2 [33]. The nature of the protein-protein interaction between IAA8 and the five TPL/TPR proteins is unknown; however, IAA8 could act as a transcriptional repressor to adjust the expression of the auxin-responsive genes according to cellular auxin levels by interacting at least with TPR2.

The transcriptional repressor Aux/IAA proteins are predicted to function in the nucleus. Aux/IAA proteins have a nuclear localization sequence (NLS) and are localized to the nucleus [18], [23], [34]–[37]. However, in contrast to IAA7 and IAA17, IAA8 is localized not only to the nucleus, but also to the cytosol (Figure 3). This distinct subcellular distribution of IAA8 was also observed in an independent study that used an *Agrobacterium*-mediated transient expression system in *Nicotiana benthamiana* [42]. IAA8 seems to lack a typical nuclear export signal sequence (data not shown). Because Aux/IAA proteins, including IAA8, possess a NLS sequence, IAA8 appears to enter the nucleus initially, and then exit to the cytosol via an unknown mechanism. Recently, IAA8 was found to interact with LSD1 (LESIONS SIMULATING DISEASE RESISTANCE 1), which negatively controls cell death and disease resistance [43]. LSD1 is a cytosolic protein that sequesters the transcription factor AtbZIP10, a positive regulator of cell death in disease resistance, in the cytosol by acting as a scaffold protein, probably to inhibit AtbZIP10 activity [44]. Thus, the function of IAA8 might also be involved in the transcriptional regulation of cell death in disease resistance, being controlled by a similar mechanism for AtbZIP10.

### IAA8 participates in the transcriptional regulation of the auxin response by interacting with TIR1 auxin receptors and ARF transcription factors in the nucleus

The abundance of Aux/IAA proteins, which is regulated by TIR1/AFB auxin receptor proteins, affects the expression of auxin-responsive genes by blocking the function of ARF transcription factors via the formation of heterodimers [5], [8]–[11]. Because a comprehensive analysis of the interaction between IAA8 and these functional partners would provide valuable insight into the functioning of the transcriptional regulation system of the auxin response, we conducted two independent protein-protein interaction assays, i.e., yeast two-hybrid analysis and bimolecular fluorescence complementation (BiFC) analysis in *Arabidopsis* mesophyll protoplasts. Auxin-dependent interactions between the TIR1 auxin receptor and IAA8 as well as the well-characterized Aux/IAA proteins, IAA7 and IAA17, were observed both in yeast and *in planta* (Figure 4). This is the first report that demonstrates the auxin-dependent physical protein-protein interaction between Aux/IAA proteins and TIR1/AFBs auxin receptors using fluorescent proteins *in planta*. It has been reported that IAA8 is degraded more gradually than other Aux/IAA proteins, such as IAA17 [20], but it remains unclear whether or not degradation of IAA8 is auxin-dependent. Our results strongly suggest that IAA8 would be degraded by the auxin-mediated interaction with TIR1/AFB receptors, which are components of the SCF^TIR1/AFB^ ubiquitin-ligase complex, like other Aux/IAA proteins in the nucleus.

Next, we conducted the same assays to examine the protein-protein interaction between IAA8 and ARF transcription factors. In yeast, IAA8 strongly interacts with the ARF activators, ARF5, ARF7, and ARF19, while the interaction levels with the ARF repressors, ARF4, ARF11, and ARF16, are much lower (Figure 5A). BiFC analysis also demonstrated that IAA8 interacts with both ARF activators and repressors even in plant cells (Figure 5B). Numerous reports suggest that *Arabidopsis* Aux/IAA proteins do not interact specifically with ARFs [18], [25], [27], [40]. There is also a report that indicates that interactions between Aux/IAAs and ARF repressors are weaker than those with ARF activators [45]. In contrast, it has recently been reported that some Aux/IAA proteins do not interact with several ARF repressors in *Arabidopsis* and rice [46], [47]. This discrepancy might be due to differences in the experimental techniques used to examine the protein-protein interaction (e.g., yeast two-hybrid assay, BiFC assay, split-luciferase assay). However, our results suggest that IAA8 preferentially interacts with ARF activators, but eventually binds to all ARF proteins in the nucleus that contain a complete domain III and IV. Because IAA8 potentially interacts with all ARF proteins *in planta*, IAA8 may participate in the transcriptional regulation of the auxin response via its interaction with ARFs expressed in the same cells, which may be identified by comparing expression profiles in a detailed cellular expression map of *Arabidopsis ARF* genes [48].

In summary, our data demonstrate that IAA8 is involved in lateral root formation and that this function appears to be regulated by interactions with the TIR1 auxin receptor and ARF transcription factors in the nucleus. The conclusion that IAA8 may have a distinct function from other Aux/IAA proteins is supported by knowledge of *IAA8* expression in response to auxin and the stability of its protein [12], [20], [28] as well as subcellular localization pattern of IAA8 (Figure 3). In addition, the phylogenetically closest homolog of *IAA8* in tomato, *IAA9*, is, in contrast to other *Aux/IAA* genes, involved in fruit development and leaf morphogenesis [49]. Therefore, further functional analysis of *IAA8*, which may encode a distinct and unique Aux/IAA protein, is required to obtain novel information about the complex mechanisms of transcriptional regulation during the auxin response. In this study, we overexpressed wild-type *IAA8*, which resulted in plants with weaker phenotypes than the gain-of-function *Aux/IAA* mutants. Considering that no gain-of-function mutations in *IAA8* have been identified by screening for plants with altered auxin responses or morphology, transgenic plants expressing *IAA8* with an artificial domain II, as found in gain-of-function mutations in *Aux/IAA* genes, which can recapitulate mutant phenotypes upon introduction into wild-type plants, are expected to produce more severe phenotypic changes and to provide novel insights into the functioning of *IAA8* in *Arabidopsis*.

## Materials and Methods

### Plant material and growth conditions

*Arabidopsis thaliana* ecotype Columbia (Col-0) was used as wild type. Seeds of *iaa8-1* [19] were obtained from the Arabidopsis Biological Resource Center (ABRC). After cold treatment for one to two days to synchronize germination, all plants were grown on soil [2∶2∶1 mixture of Supermix A (Sakata seed, Japan), vermiculite, perlite] under controlled environmental conditions at 12 h light/12 h dark cycles at 22°C.

### Plasmid construction and *Arabidopsis* transformation

To create the *XVE::IAA8* construct, which consists of *IAA8* driven by an estrogen-inducible promoter, XVE, in the pER8 vector [30], the *Arabidopsis IAA8* cDNA fragment was amplified by PCR with gene-specific primer sets (see Table S1) and cloned into pDONR207 (Invitrogen), using the Gateway BP recombination method (Invitrogen). After verifying the nucleotide sequence of the PCR fragment by sequencing, the *IAA8* cDNA fragment was transferred into the modified pER8 estradiol-inducible plant transformation vector [30], into which the Gateway cassette had been inserted using the Gateway Vector Conversion System, and the *bar* gene, for selection of transgenic plants, using LR clonase (Invitrogen), according to the manufacturer's instruction (Invitrogen). The resultant vector was introduced into *Agrobacterium tumefaciens* strain GV3101 (pMP90) by electroporation. The transformed *A. tumefaciens* was used for floral dip transformation of *Arabidopisis* Col-0 as described in [50]. Transgenic plants were selected on soil by spraying with diluted commercial BASTA solution (Bayer Japan) as described in [51].

### Phenotypic analysis of *Arabidopsis* roots

All seeds were surface sterilized in 50% commercial bleach and 0.01% Silwet L-77 (Toray DowCorning), subjected to cold treatment, and then vertically grown on half strength Murashige and Skoog (MS) medium supplemented with 1% sucrose under the same conditions as for growth in soil. To monitor root growth and lateral root formation, seedlings were grown for 14 days. The length of primary roots and the number of lateral roots were determined for at least 20 seedlings in each genotype. The gravitropism assays were carried out according to Park *et* *al.* [31].

### RNA isolation and semi-quantitative RT-PCR

The roots of two-week-old plants grown on half strength MS medium as described above were immersed in 10 μM β-estradiol for 24 h (estrogen treatment) and then transferred to 1 μM indole-3-acetic acid (IAA) solution (auxin treatment). Total RNA was isolated using Total RNA Extraction Kit Mini (Plant) (RBC Bioscience). First-strand cDNA was synthesized from 1 μg of total RNA treated with DNase I (TAKARA BIO) using the PrimeScript II 1st strand cDNA Synthesis Kit (TAKARA BIO). PCR amplification was then performed using GoTaq Green Master Mix (Promega). The gene-specific primers and PCR cycles for each gene are listed in Table S1.

### Yeast two-hybrid analysis

The fragments of *IAA7* and *IAA17* cDNAs and the C-terminal domain (CTD) fragments of *ARF3*, *ARF4*, *ARF5*, *ARF7*, *ARF11*, *ARF16,* and *ARF19* cDNAs were amplified by PCR using plasmids harboring full-length *Aux/IAA* and *ARF* cDNAs from RIKEN *Arabidopsis* cDNA Encyclopedia DNABook [52] as template DNAs, and then cloned into pDONR221 or pDONRzeo (Invitrogen) using BP Clonase II (Invitrogen). The gene-specific primers for PCR are listed in Table S1. After verifying the nucleotide sequence of PCR fragments by sequencing, the *IAA8* cDNA fragment was transferred into bait plasmid vector pEG202gw, and *IAA7*, *IAA17,* and *ARFCTD* fragments were cloned into prey plasmid vector pJG4-5gw [53], respectively, using LR clonase II (Invitrogen). The Gateway-compatible SSP gold standard full-length cDNA clone [54] of *TIR1* (GC105370) was obtained from ABRC and used for transferring fragments into pEG202gw, as described above. A yeast two-hybrid assay using the LexA-based two-hybrid system was basically carried out as described in [44]. Briefly, the transformation of EGY48 yeast cells (*MATα ura3 trp1 his3 3LexAop-LEU2*) harboring pJK103 [*2LexAop-lacZ*]) reporter plasmid was carried out with the Frozen-EZ Yeast Transformation II Kit (Zymo Research). The strength of interaction between IAA8 and each ARFCTD was evaluated by measuring β-gal activity using the *ο*-Nitrophenyl-β-D-galactopyranoside (ONPG) method, according to the Yeast Handbook (Clontech). To test for interactions between TIR1 and Aux/IAAs, transformants with both TIR1 in pEG202 and Aux/IAAs in pJG4-5 were transferred onto SD(Gal)/-Ura/-His/-Trp/-Leu with 100 μM indole-3-acetic acid (IAA). All plates were incubated for 2–3 days at 30°C.

To confirm the expression levels of IAA8 and ARFCTD proteins co-expressed in yeast, the extracted total protein from each transformant was subjected to SDS-PAGE and then transferred onto Protoran nitrocellulose membrane (GE Healthcare) for Western blot analysis. Rabbit anti-LexA (BioAcademia) and rat anti-HA (3F10; Roche) antibodies were used for the detection of LexA DNA-binding domain fusion of IAA8 and activation domain with HA tag fusion of each ARFCTD, respectively. Luminata Crescendo Western HRP substrate (Millipore) was used for chemiluminescent detection.

### Plasmid Construction for GFP fusions and BiFC analysis

For the construction of *IAA7-*, *IAA8-* and *IAA17-GFP* fusions driven by the CaMV 35S promoter, all IAA cDNA fragments made as described above were transferred into p2GWF7 [55], using LR Clonase II (Invitrogen). Similarly, for the construction of nYFP or cYFP fusion genes, which were driven by the CaMV 35S promoter for BiFC experiments, full-length cDNAs of *ARF3*, *ARF4*, *ARF5*, *ARF7*, *ARF11*, *ARF16,* and *ARF19* were amplified by PCR using plasmids in the RIKEN *Arabidopsis* cDNA Encyclopedia DNABook [52] as template and cloned into pDONRzeo using the Gateway BP recombination reaction. The gene-specific primers for PCR are listed in Table S1. After verifying the nucleotide sequence of PCR fragments of ARF full-length cDNAs by sequencing, *nYFP-Aux/IAAs*, *ARFs-nYFP, cYFP-TIR1,* and *IAA8-cYFP* fusions driven by the CaMV 35S promoter were constructed by transferring *Aux/IAA, ARF, TIR1,* and *IAA8* full-length cDNAs into nYFP/pUGW0, nYFP/pUGW2, cYFP/pUGW0, and cYFP/pUGW2 [56], respectively, using the Gateway LR recombination reaction. As a negative control, nYFP-GUS driven by the CaMV 35S promoter was also created using nYFP/pUGW0 and pENTR-gus (Invitrogen), as described above. To create NLS-tdTomato, which was used as a nuclear organelle marker and a control for transformation, the amplified fragment of the simian virus 40 (SV40) large T antigen nuclear localization signal (NLS) [38] was cloned behind the CaMV 35S promoter into pDONRzeo (Invitrogen) and then transferred into pGWtd [57] using the Gateway recombination method.

### Transient expression in *Arabidopsis* mesophyll protoplasts and confocal microscopy

Mesophyll protoplasts from the leaves of four-week-old *Arabidopisis* Col-0 plants grown on soil were prepared and transformed using the PEG-calcium transfection method [58]. Protoplasts co-transfected with 5 μg of GFP-fusion plasmid or 10 μg of nYFP- and cYFP-fusion plasmids for BiFC analysis and 1 μg of NLS-tdTomato plasmid were assayed for fluorescence 20–24 h after transfection using a confocal laser scanning microscope (Fluoview FV10i-O; Olympus). To evaluate the TIR1-IAA interaction by BiFC analysis, 10 μM IAA was added to the transfected protoplast solution 30–60 min before microscopic observation. The fluorescence signals from GFP, YFP, and tdTomato were excited by 489-, 480-, and 580-nm wavelengths, respectively, and emissions were observed at 510-, 527-, and 610-nm wavelengths, respectively. The data were exported as 8-bit TIFF files and processed using Adobe Photoshop CS5 (Adobe Systems).

## Supporting Information

Figure S1 **The primary root length of Col-0,** ***XVE::IAA8*** **transgenic plants, and the** ***iaa8-1*** **mutant.** All seedlings were vertically grown for two weeks on 1/2 MS medium containing 10 μM β-estradiol (+β-estradiol) or 0.1% ethanol (−β-estradiol) and then primary root length was measured. The averages of at least 20 seedlings ± S.D. are shown.
(EPS)

Figure S2 **The phenotype of wild-type (Col-0) and** ***IAA8*** **loss-of-function mutant (** ***iaa8-1*** **) seedlings.** All seedlings were vertically grown for two weeks on 1/2 MS medium containing 10 μM β-estradiol (+β-estradiol). Bar  = 1 cm.
(EPS)

Figure S3 **Western blot analysis of IAA8 and ARF proteins co-expressed in yeast.** BD-IAA8 and AD-ARFCTD expressed in each yeast transformant as shown in Figure 5A were detected using anti-LexA and anti-HA antibodies, respectively. White arrowheads indicate the detected bands corresponding to predicted molecular weight for each AD-ARFCTD protein.
(EPS)

Table S1 **Nucleotide sequences of primers used in this study.**
(XLSX)
